The article "Changes of Intestinal Flora and Lymphocyte Subsets in Patients with Chronic Renal Failure" was retracted in 2023. Reasons: signs of a paper mill; compromised peer review; unreliable results or conclusions.

# Changes of Intestinal Flora and Lymphocyte Subsets in Patients with Chronic Renal Failure

**DOI:** 10.1155/2021/4288739

**Published:** 2021-10-15

**Authors:** Yan Lv, Gang Ren, Xiaojun Ren

**Affiliations:** ^1^Department of Nephrology, Shanxi Bethune Hospital, Shanxi Academy of Medical Sciences, Tongji Shanxi Hospital, Third Hospital of Shanxi Medical University, Taiyuan 030032, China; ^2^Department of Neurology, Shanxi Bethune Hospital, Shanxi Academy of Medical Sciences, Tongji Shanxi Hospital, Third Hospital of Shanxi Medical University, Taiyuan 030032, China

## Abstract

**Objective:**

To explore the changes of intestinal flora and lymphocyte subsets in patients with chronic renal failure (CRF).

**Methods:**

60 CRF patients who were treated from June 2018 to June 2019 were selected; 60 healthy persons were selected as the control group. 16S rDNA was used to detect the expression of *Lactobacillus*, Enterobacteriaceae, *Enterococcus*, *Bacteroides*, *Clostridium,* and *Bifidobacterium* in the feces of the two groups. Illumina Miseq sequencing (Solexa sequencing technology) method was used to analyze the structural differences and species diversity of intestinal flora, including species richness index (Chao) and diversity index (Shannon, Simpson). Flow cytometry was used to detect the levels of lymphocytes and their subgroups of the two groups. Pearson correlation analysis was used to analyze the correlation between Chao and lymphocyte subsets.

**Results:**

The number of Enterobacteriaceae and *Enterococcus* in CRF group were higher than those in the control group (*P* < 0.05), while the *Lactobacillus*, *Bacteroides*, *Clostridium,* and *Bifidobacterium* were opposite (*P* < 0.05). The Simpson index of the CRF group was lower than that of the control group, while the Chao index and Shannon index were opposite (*P* < 0.05). The levels of CD3^+^, CD4^+^, CD8^+^, and CD4^+^/CD8^+^ in the CRF group were lower than those in the control group, while the levels of CD14^+^, CD19^+^, and CD16^+^/CD56^+^ were opposite (*P* < 0.05). The intestinal flora Chao index of CRF group was negatively correlated with the levels of CD3^+^, CD4^+^, and CD8^+^ (*r* = −0.692, *P*=0.019; *r* = −0.669, *P*=0.021; *r* = −0.603, *P*=0.028). The intestinal flora Chao of CRF group is positively correlated with the level of CD14^+^ and CD16^+^/CD56^+^ (*r* = 0.615, *P*=0.026; *r* = 0.758, *P*=0.016).

**Conclusion:**

There are intestinal flora disorder and the imbalance of immune function in CRF patients, which are mainly manifested in the change of intestinal flora structure, the increase of richness and diversity of intestinal flora, and the decrease of lymphocyte subgroups. There is correlation between the imbalance of intestinal colony and the imbalance of immune function.

## 1. Introduction

Chronic renal failure (CRF) is a clinical syndrome that causes chronic and substantial damage to the kidneys caused by primary glomerulonephritis, chronic pyelonephritis, hypertension, and renal arteriosclerosis, which in turn leads to a decline in renal function [1]. The prevention and treatment of CRF have become an important public health problem faced by countries all over the world. Finding effective methods, delaying the process, improving quality of life, and prolonging survival are important contents of the prevention and treatment of CRF, which has important clinical significance. CRF patients need to limit salt and water, high-quality low-protein diet, iron supplementation, and anti-infective treatment to deal with prone to anemia and infection, which can cause changes and imbalance of intestinal flora and interfere with the intestinal absorption of nutrients [2]. The main causes of death in CRF patients are severe infections and cardiovascular diseases. Among them, CRF deaths due to severe infections account for 13.1% to 35.7%, and immune function imbalance is one of the main causes of severe infections in CRF patients [3]. In this study, the intestinal flora composition and lymphocyte subpopulation levels of CRF patients and normal people were compared to explore the changes and correlations of the intestinal flora and lymphocyte subpopulations of CRF patients. The specific research is as follows.

## 2. Object and Methods

### 2.1. Research Object

60 CRF patients who were treated in our hospital from June 2018 to June 2019 were selected as the CRF group. Among them, 36 were females and 24 were males, aged from 28 to 65 years old, with an average age of (41.32 ± 8.76) years old. 60 healthy people undergoing physical examinations at the same period were selected as the control group. Among them, 28 were females and 32 were males, aged from 27 to 63 years, with an average age of (42.76 ± 9.16) years. There was no significant difference in gender and age between the two groups (*P* > 0.05). Inclusion criteria: meet the CRF diagnostic criteria [4]. Exclusion criteria: (1) suffering from intestinal disease. (2) Taking immune-related drugs or receiving immunotherapy within 3 months. (3) Suffering from severe infection. (4) Having taken antibiotic drugs recently. This study was reviewed and approved by the ethics committee of our hospital, and all patients or their family signed the informed consent form.

### 2.2. Methods

#### 2.2.1. Intestinal Flora Structure Detection

Stool samples were collected and placed in a stool collector within 2 hours after defecation of all subjects and then stored in a refrigerator at −80°C. According to the product manual of TIANamp Stool DNA Kit (TIANGEN), 200 mg of each stool sample was weighed, genomic DNA was extracted, and it was stored at −20°C. The purity and concentration of DNA were then detected by agarose gel electrophoresis, and an appropriate amount of sample DNA was placed in a centrifuge tube and diluted to 1 mg/L with sterile water. PCR was performed using diluted genomic DNA as a template, bacteria-specific primers for *Lactobacillus*, Enterobacteriaceae, *Enterococcus*, *Bacteroides*, *Clostridium,* and *Bifidobacterium* were designed, and sequence specificity comparisons were performed in the BLAST gene library primers, as shown in Table 1. Amplified regions included 16S rDNA V3-V4. The library was constructed using TruSeq DNA PCR-Free Sample Preparation Kit. The constructed library was quantified by Qubit and Q-PCR. Once qualified, high-throughput sequencing was performed using NovaSeq6000.

#### 2.2.2. Detection of Intestinal Flora Richness and Diversity

Illumina Miseq high-throughput sequencing method (Solexa sequencing technology) was used to detect the intestinal flora sequence (Shanghai Lingen Biotechnology Company), and high-quality sequences were extracted, and OTU cluster analysis and species taxonomy analysis were performed on them, and the diversity index and flora structure were analyzed. The diversity analysis (Alpha diversity) of a single sample reflects the abundance and diversity of the microbial community; the I-Sanger biological information analysis platform (http://www.i-Sanger.com/) of MGB was used for the diversity analysis of intestinal flora. The Chao index is used to calculate the richness of the flora. The Chao index is commonly used in ecological research to estimate the total number of species. The Shannon and Simpson indexes are used to calculate the diversity of the flora. The higher the Shannon index, the higher the diversity of the flora, and the higher the Simpson index, the lower the diversity of the flora [5].

#### 2.2.3. Detection of Lymphocyte Subgroups

Fasting venous blood was taken from CRF patients and normal control group for examination. The 201 fluorescein-labeled monoclonal antibody was put into a 16X-75 Falcon capped sample tube (BD Company), and then 100 *μ*l heparin anticoagulated whole blood was add, mixed well, and kept in the dark at room temperature for 20 minutes; 100 *μ*l of hemolysin was added, mixed well, and placed in the dark at room temperature for 10 minutes; 500 *μ*l of 1% paraformaldehyde-containing PBS was added to fix the cells, they were stored in a dark place at 2°C to 8°C, and a flow cytometer (FACSCalibur Flow Cytometer, BD Company) was used to detect them. In order to ensure that there are at least 4000 lymphocytes in the lymphocyte gate, the CellQuest software is used to obtain and analyze the cells.

### 2.3. Statistical Methods

The SPSS19.0 software was used for data processing, the measurement data were expressed as mean ± standard deviation (mean ± SD), and the pairwise comparison was analyzed by *t*-test. The enumeration data were expressed by (%), and the comparison between groups was analyzed by *χ*^2^ test. Correlation analysis adopts Pearson correlation analysis. The test level is *α* = 0.05, and *P* < 0.05 indicates that the difference is statistically significant.

## 3. Results

### 3.1. Comparison of Intestinal Flora between the Two Groups

The number of Enterobacteriaceae and *Enterococcus* in CRF group were higher than those in the control group, and the number of *Lactobacillus*, *Bacteroides*, *Clostridium,* and *Bifidobacterium* were lower than those in the control group; the difference was statistically significant (*P* < 0.05), as shown in Figure 1.

### 3.2. Comparison of Intestinal Flora Richness and Diversity

The Simpson index of the CRF group was lower than that of the control group, the Chao index and Shannon index of the CRF group were higher than those of the control group, and the difference was statistically significant (*P* < 0.05), as shown in Figures 2–4.

### 3.3. Analysis of Changes in Lymphocytes Subgroups

The levels of T lymphocytes (CD3^+^), CD4^+^, CD8^+^, and CD4^+^/CD8^+^ ratios in the CRF group were lower than those in the control group, the levels of monocytes (CD14^+^), B lymphocytes (CD19^+^), and NK cells (CD16^+^/CD56^+^) were higher than those in the control group, and the differences were statistically significant (*P* < 0.05), as shown in Figures 5 and 6.

### 3.4. Correlation Analysis between the Richness of Intestinal Flora and the Changes of Lymphocyte Subgroups

The richness of intestinal flora in the CRF group was negatively correlated with the levels of T lymphocytes (CD3^+^), CD4^+^, and CD8^+^ (*r* = −0.692, *P*=0.019; *r* = −0.669, *P*=0.021; *r* = −0.603, *P*=0.028). The richness of intestinal flora in the CRF group was positively correlated with the levels of monocytes (CD14^+^) and NK cells (CD16^+^/CD56^+^) (*r* = 0.615, *P*=0.026; *r* = 0.758, *P*=0.016), as shown in Figures 7–11.

## 4. Discussion

There are more than 1,000 kinds of bacteria in healthy human intestines, which constitute a huge and complex human digestive tract microbial system [6]. Intestinal flora is a type of microorganisms that coexist with humans. It participates in the absorption and metabolism of nutrients and the synthesis of important substances, maintains intestinal health, and induces the maturation and tolerance of the immune system. Changes in the composition, richness, and functional gene differences of the intestinal microbial system are closely related to health and disease of humans [7]. CRF causes intestinal flora imbalance due to various reasons, and the resulting intestinal urinary toxins and endotoxins promote the progress of CRF and the occurrence of complications [8].

Enterobacteriaceae and *Enterococcus* belong to harmful bacteria, and *Lactobacillus*, *Bacteroides*, *Clostridium,* and *Bifidobacterium* belong to beneficial bacteria. The increase of intestinal richness represents the increase of pathogenic bacteria in the intestinal tract. The results of this study showed that the number of Enterobacteriaceae and *Enterococcus* in the CRF group were higher than those in the control group, while the *Lactobacillus*, *Bacteroides*, *Clostridium,* and *Bifidobacterium* were opposite, which is similar to the study by Syed-Ahmed et al. [9]. Besides, the Simpson index of the CRF group was lower than that of the control group, while the Chao index and Shannon index were opposite. The results show that the structure of the intestinal flora has changed significantly, and the abundance and diversity of the intestinal flora have increased in patients with CRF. The main reasons leading to the imbalance of the intestinal flora of CRF patients include the following points: (1) with the aggravation of renal damage in patients with CRF, the number and types of intestinal bacteria gradually increase and bacteria overproduce, which lead to the production of a large number of opportunistic pathogens [10]. (2) With the decline of renal function in patients with CRF, a large amount of uric acid and oxalic acid are actively secreted from the intestinal epithelium to the intestinal cavity, which change the energy metabolism of the intestinal flora [11]. (3) Because CRF patients need to limit the intake of salt and water and a high-quality low-protein diet, the intake of potassium ions and dietary fiber such as fruits and fresh vegetables are reduced, and the ratio of intestinal fiber to protein is imbalanced, which leads to a decrease in the proportion of hydrolyzable protein of *Clostridia* and *Bacteroides* [12]. (4) The increased risk of infection and the accompanying renal anemia have led to an increase in the frequency of antibiotic and iron use in patients with CRF, which will also lead to changes in the structure of the intestinal flora [13]. In addition, the imbalance of intestinal flora can further cause immune system diseases, leading to the deterioration of CRF [14].

CRF patients are prone to infection, mainly due to the defect of lymphocyte function, especially T lymphocyte function; their number of lymphocytes that mediate the human immune response continues to decrease, accompanied by T cell dysfunction [15]. The role of CD4^+^ T cells mainly includes enhancing cell-mediated immune responses, promoting the proliferation and differentiation of B cells (CD19^+^) and helping to produce antibodies that participate in humoral immune responses [16]. CD8^+^ T cells can specifically kill tumor cells and tissue cells infected by pathogenic microorganisms and inhibit cellular and humoral immunity. CD4^+^ cells and CD8^+^ cells jointly regulate cellular and humoral immunity, exerting anti-infection and antitumor effects. The results of this study show the levels of CD3^+^, CD4^+^, CD8^+^, and CD4+/CD8+ in the CRF group were lower than those in the control group, which indicates that patients with CRF have decreased lymphoid subpopulation cell levels and immune function imbalance. The reason may be related to the increase of CRF toxin, parathyroid hormone, iron load, prostaglandin E2, and muscle derivatives, especially methyl muscle [17]. In addition, this study also found that monocytes (CD14^+^), B cells (CD19^+^), and NK cells (CD16^+^/CD56^+^) increased significantly compared with the normal population. At present, the specific mechanism of this situation is not clear, and it is mostly believed that it may be a compensation mechanism for the decrease in the number of lymphocytes required for the specific immune function of CRF patients [18, 19].

In addition, Pearson correlation analysis shows the richness of intestinal flora was negatively correlated with the levels of CD3^+^, CD4^+^, and CD8^+^ and positively correlated with the levels of CD14^+^ and CD16^+^/CD56^+^. The reason may be that the imbalance of the intestinal flora destroys the homeostasis of the intestinal microenvironment, causing lymphocytes to accumulate in the intestines and the excessive production of prooxidation, proinflammatory, and other harmful metabolites [20, 21]. CD3^+^, CD4^+^, and CD8^+^ cells are closely related to the body's immunity. When the immunity is low, their expression will be decreased. Monocytes and NK cells are closely related to the body's inflammatory reaction. When the body's inflammatory injury is aggravated, their expression will be increased. In patients with CRF, their immune function will be decreased, and the intestinal microflora will be increased, accompanied by the aggravation of inflammatory injury. Hence, Chao has a negative correlation with cells such as CD3^+^, but a positive correlation with monocytes.

## 5. Conclusion

There are intestinal flora disorder and the imbalance of immune function in CRF patients, which are mainly manifested in the change of intestinal flora structure, the increase of richness and diversity of intestinal flora, and the decrease of lymphocyte subgroups. There is correlation between the imbalance of intestinal colony and the imbalance of immune function.

## Figures and Tables

**Figure 1:** Quantitative PCR results when intestinal bacteria are implemented. Note: comparison of the same index between the two groups, *P* < 0.05.

**Figure 2:** Comparison of Chao index. Note: comparison between the two groups, *P* < 0.05.

**Figure 3:** Comparison of Shannon index. Note: comparison between the two groups, *P* < 0.05.

**Figure 4:** Comparison of Simpson index. Note: comparison between the two groups, *P* < 0.05.

**Figure 5:** Comparison of CD3^+^, CD4^+^, CD8^+^, CD14^+^, and CD19^+^. Note: comparison of the same index between the two groups, *P* < 0.05.

**Figure 6:** Comparison of CD4^+^/CD8^+^ and CD16^+^/CD56^+^. Note: comparison of the same index between the two groups, *P* < 0.05.

**Figure 7:** Correlation analysis between the Chao index and the CD3+.

**Figure 8:** Correlation analysis between the Chao index and the CD4+.

**Figure 9:** Correlation analysis between the Chao index and the CD8+.

**Figure 10:** Correlation analysis between the Chao index and the monocytes (CD14+).

**Figure 11:** Correlation analysis between the Chao index and the NK cells (CD15+/CD56+).

**Table 1:** Primer information.

Bacteria	Primer	Primer sequence	Annealing temperature (°C)	Sequence length (bp)
*Lactobacillus*	g-Lacto-F	5′-AGCAGTAGGGAATCTTCCA-3′	58	341
	g-Lacto-R	5′-CACCGCTACACATGGAG-3′		

Enterobacteriaceae	g-Esche-F	5′-GTTAATACCTTTGCTCATTGA-3′	58	340
	g-Esche-R	5′-ACCAGGGTATCTAATCCTGTT-3′		

*Enterococcus*	g-Enter-F	5′-CCCTTATTGTTAGTTGCCATCATT-3′	52	140
	g-Enter-R	5′-ACTCGTTGTACTTCCCATTGT-3′		

*Bacteroides*	g-Bfra-F	5′-ATAGCCTTTCGAAAGRAAGAT-3′	60	501
	g-Bfra-R	5′-CCAGTATCAACTGCAATTTTA-3′		

*Clostridium*	g-Ccoc-F	5′-AAATGACGGTACCTGACTAA-3′	60	438–441
	g-Ccoc-R	5′-CTTTGAGTTTCATTCTTGCGAA-3′		

*Bifidobacterium*	g-Bifid-F	5′- CTCCTGGAAACGGGTGG-3′	58	549–563
	g-Bifid-R	5′-GGTGTTCTTCCCGATATCTACA -3′		

## Data Availability

The data are available from the corresponding author.
